# Sustainability and Environmental Impact of Ethanol and Oxyhydrogen Addition on Nanocoated Gasoline Engine

**DOI:** 10.1155/2022/1936415

**Published:** 2022-01-20

**Authors:** Sambandam Padmanabhan, K. Giridharan, Balasubramaniam Stalin, V. Elango, J. Vairamuthu, P. Sureshkumar, Leta Tesfaye Jule, Ramaswamy Krishnaraj

**Affiliations:** ^1^School of Mechanical and Construction, Vel Tech Rangarajan Dr. Sagunthala R&D Institute of Science and Technology, Chennai 600062, Tamil Nadu, India; ^2^Department of Mechanical Engineering, Easwari Engineering College, Chennai 600089, Tamil Nadu, India; ^3^Department of Mechanical Engineering, Anna University, Regional Campus Madurai, Madurai 625019, Tamil Nadu, India; ^4^Department of Mechanical Engineering, Sethu Institute of Technology, Pulloor Kariapatti, Virudhunagar 626115, Tamil Nadu, India; ^5^Department of Mechanical Engineering, Ramco Institute of Technology, Rajapalayam 626117, Tamil Nadu, India; ^6^Centre for Excellence-Indigenous Knowledge, Innovative Technology Transfer and Entrepreneurship, Dambi Dollo University, Dambi Dollo, Ethiopia; ^7^Department of Physics, College of Natural and Computational Science, Dambi Dollo University, Dambi Dollo, Ethiopia; ^8^Department of Mechanical Engineering, Dambi Dollo University, Dambi Dollo, Ethiopia

## Abstract

Climate change, clean air, renewable energy, nontoxic surroundings, and the opportunity to live in a healthy community are just few of the issues that environmental sustainability addresses. To improve environmental health and quality of life, several researchers have turned their attention to alternative energy sources like ethanol and oxyhydrogen. In latest years, significant progress has been made in the development of ethanol and hydrogen as clean energy sources. A higher octane rating is achieved by mixing ethanol with gasoline rather than using regular gasoline. A novel mix of oxyhydrogen, ethanol, and gasoline is ecologically friendly while simultaneously increasing the performance of gasoline engines. In this study, a nanoparticle-coated piston on a low heat rejection gasoline engine fuelled by an ethanol-gasoline mix with oxyhydrogen addition was investigated. It has been evaluated that thermal efficiency improved by up to 25% while fuel consumption can be reduced by up to 28% on a volume basis compared to the baseline engine. Furthermore, the decrease in harmful carbon monoxide reached around 10%, and the reduction in unburned hydrocarbon emissions reached 18%.

## 1. Introduction

The researchers conducted a study on the burning of ethanol in an internal combustion engine. To improve performance and thermal efficiency, the utilization of high compression hydrous ethanol reforming and supercharging lean-burn circumstances was investigated [1]. The addition of ethanol to gasoline increased nitrogen oxides (NOx) emissions. Hydrocarbon (HC) and carbon monoxide (CO) emissions are reduced in aggregate. It was found that differing ethanol-to-gasoline blend ratios resulted in varying degrees of energy efficiency and pollution under a variety of loading conditions. The findings indicated that emission concentrations rose as engine load increased but reduced as ethanol content increased [2]. The impact of a mix of ethanol and gasoline on power, torque, fuel consumption, and emissions was investigated using analytically assessed steady-state engines [3]. The majority of gasoline-ethanol blends research in engines to date has been on ethanol mix percentages up to twenty percent, with variable degrees of success. The results of several experiments showed little or no response to ethanol concentration up to 10% by volume, suggesting that engine operating circumstances have a more significant impact on engine characteristic and emissions at low-ethanol blend levels. Recent attention has focused on the performance of spark-ignition (SI) engines running on ethanol-gasoline mixes with a constant fuel-air ratio [4, 5]. As engine speed increases and the proportion of ethanol in the fuel mix decreases, volumetric efficiency tends to decline. Substantial reduction in exhaust gas emissions occurs when ethanol ratios are increased in comparison to gasoline fuel [6]. Saturated HC emissions such as methane and ethane increased as ethanol blends were increased over 20%. More aromatics and unburned ethanol emissions were created by higher ethanol blends than straight gasoline and mixtures. All emissions components were reduced as vehicle speed increased [7]. This is due to the fact that ethanol contains a higher concentration of oxygen atoms. The gasoline requires a greater quantity of oxygen to burn, displaying more reputation between 10 and 15% of ethanol blends, which may reduce emissions completely. Fuels with a greater ethanol content offered a significant emissions advantage over conventional fuels [8]. The purpose of this study is to examine the feasibility of dual-fuel operation in gasoline engines employing acetone, butanol, ethanol, and hydroxy gas enrichment. Dual-fuel operation resulted in considerable CO, HC, and smoke reductions. Carbon dioxide and nitrogen oxides emissions, on the other hand, increased when combustion oxidation was increased and combustion temperatures were increased [9]. Hydrous ethanol is cheaper and uses less energy to produce than anhydrous ethanol. The water ratio in ethanol impacts the energy consumption in ethanol manufacturing. Hydrous ethanol enhanced flame growth and propagation time, but not flame stability [10]. The homogenous and stable gasoline-methanol-ethanol combination was tested. In all engine settings, a low-methanol mix provides more power than pure gasoline [11]. Because ethanol-gasoline and methanol-gasoline mixtures have different characteristics, the combustion system is altered. Due to these factors, it is difficult to pinpoint the principles of how ethanol or methanol impacts emissions [12]. Low-ethanol mixes with less than 20% ethanol had no obvious effect on engine efficiency or torque, but the performance of the engine decreased when the proportion of blending was increased [13]. A higher heat of vaporization is produced by ethanol fuel as compared to conventional gasoline. As a result, the temperature peak within the cylinder is reduced, and the engine power is increased.

Oxyhydrogen is one of the alternative energy sources that may be utilized in place of fossil fuels. Electrolysis of water may be used to produce it in certain circumstances. Oxyhydrogen boosts the engine's power and thermal efficiency while minimizing the development of harmful carbon deposits, nitrogen oxides, and hydrocarbons. Numerous researchers [14, 15] are investigating oxyhydrogen as a possible engine enhancer for gasoline and diesel engines and for other power source applications. A mixture of oxyhydrogen, air, and gasoline reduced pollutant emissions and improved engine efficiency significantly [16]. The proprietary mix was evaluated at a variety of engine speeds. Nitrogen oxide emissions were almost halved. Additionally, CO emissions were found to be lowered by 20% and fuel consumption was reduced by 25% [17]. The researchers experimented with different hydrogen concentrations. They found that, regardless of the hydrogen concentration, the CO emission rate remained constant and that the hydrogen concentration may control the particle emission size [18]. The gasoline engine is injected with oxyhydrogen, and the amount of gas used varies according to the available supply. Under oxyhydrogen, specific fuel consumption (SFC) and brake thermal efficiency (BTE) were increased [19]. A thorough evaluation of hydrogen mixed with improved natural gas was published, concluding an experimental investigation of hydrogen-natural gas [20]. Configurations of oxygen-hydrogen gas generators are examined. Numerical studies on the manufacturing of oxyhydrogen gas are also studied. The usage of oxyhydrogen gas in IC engines was discussed [21]. The addition of oxyhydrogen to gasoline and diesel engines increases the cleanliness of exhaust gases at idle. The amounts of CO and HC in the exhaust gases were lowered. At idle, the concentration of NOx in diesel engines rises whereas it falls in gasoline engines [22]. Oxyhydrogen flow rates of 0.5 and 0.75 LPM were generated by dry and wet cells, respectively. The addition of oxyhydrogen gas increased thermal efficiency by 20%. CO, HC, and smoke emissions were reduced in both dry and wet cells. The addition of oxygen-hydrogen gas resulted in a 42% rise in NOx emissions. The combustion properties of both dry and wet designs improved [23]. The use of oxygen-enriched diesel increases torque and power output significantly. The engine efficiency of biodiesel enhanced with oxygen is reduced with a 5% improvement in fuel consumption and thermal efficiency [24].

Several researchers are constantly developing innovative methods to improve the characteristics of the diesel engine via component change. Thermal barrier coating on components of combustion chamber is one of the most effective ways to prevent heat build-up within the chamber, resulting in improved combustion. To resist the heat shock generated during combustion, coating materials should have a high coefficient of thermal expansion [25]. Thermal barrier coatings on engines are referred to as low heat rejection (LHR) engines since they reduce heat rejection and recover combustion energy. On the combustion of biodiesel in combustion chamber components that were covered with a temperature robust ceramic substance, the particular fuel consumption rose with blended diesel and coated applications, although it decreased at low speeds when using low heat rejection diesel and mixed diesel. Copper and cadmium nanocatalyst coated pistons were used to reduce emissions while researching a diesel engine. The findings showed a significant reduction in nitrogen oxides emissions, CO emissions, and hydrocarbon emissions when a coated piston was used [26]. The effects of waste cooking palm oil on the performance of a thermal barrier coated compression ignition (CI) engine: when using waste cooking palm oil blends, the coated engine had greater fuel consumption and worse efficiency than the uncoated engine [27]. On a partly insulated single-cylinder SI engine, experimental research is carried out to study the emission characteristics and performance when the engine is fuelled with two different mixes of butanol and gasoline, respectively [28].

Small gasoline engines, which are still extensively utilized in India and produce significant levels of pollution, are still prevalent. Since renewable energy is not available in all places and seasons across India, various adjustments are required to increase the combustion rate and thermal efficiency. It is generated from agricultural resources such as sugarcane and maize; it is a feasible alternative to gasoline in terms of decreasing reliance upon foreign oil and net carbon emissions from the transportation sector. It has the potential to improve the performance of a light-duty gasoline-powered generator engine. Completing the combustion of oxyhydrogen with gasoline reduces the amount of hazardous pollutants released. An experimental investigation was carried out on a gasoline engine with a nanoparticle coating on the piston. Ten percent, fifteen percent, and twenty percent ethanol blended gasoline fuels are used to produce tertiary fuel blends, with 0.07 g/sec oxyhydrogen being added on top. The required test runs were carried out under four distinct load situations ranging from 25% to full load in order to guarantee the best possible performance and the lowest possible pollutant emissions. The goal of this research is to optimize the interdependent response of the air-fuel supply, as well as the addition of oxyhydrogen and ethanol. A complete fractional design is utilized to establish the optimal operating state that will be employed in future operations. The results are compared to those obtained using base gasoline and then evaluated utilizing a full fractional design on the design of experiments.

## 2. Materials and Methods

It reduces heat loss during combustion and therefore improves thermal efficiency in diesel engines. Because of the need to meet pollution standards while conserving gasoline, ceramic insulating methods are gaining traction. Thermal barrier coatings comprise a ceramic topcoat on top of the metal substrate and bond coating. Ceramic materials must have high thermal expansion coefficients and Poisson's ratios to operate effectively at higher combustion temperatures. They should also be thermally inert and have a stable phase.

The various studies on nanocoating materials and thickness are presented in Table 1. The coating was created using a plasma spray coating process and a distinct mix ratio of yttria-stabilized zirconia, aluminium oxide, and silicon oxide. The trial findings demonstrated superior exhaust emission reductions when compared to other blend-coated pistons optimized using genetic algorithm and neural network [35]. Numerical analyses of a gasoline homogenous charge compression ignition lean-burn engine were studied. Under the higher mechanical strength situation, increased peak cylinder pressure of 400 bar might improve BTE by more than 50% [36]. The effects of a thin thermal barrier coating layer were created on the piston crown utilizing the Micro-arc oxidation technology on the engine characteristics of a port fuel gasoline engine. The combustion flames of coated and uncoated piston engines were compared using an endoscopic imaging approach [37]. Several researchers have used plasma spray coating, one of several coating methods, to decrease heat loss from high-temperature environments [29–34]. Initially, a 200 *μ*m thick nickel chromium aluminium yttrium bond coating was put to the top crown of the aluminum alloy piston, and a 300 *μ*m thick zirconia ceramic coating was applied to surface of the piston.

Due to the global energy crisis, hydrogen is the most dependable option. Electrolysis is useful for producing hydrogen. Oxyhydrogen is still used in water-powered vehicles. Despite the enormous amount of energy needed to break down water molecules, oxyhydrogen fuel additives remain contentious. This study uses titanium electrodes as both cathode and anode to electrolyze water to produce oxyhydrogen. In an electrolytic cell, sodium sulphate decomposes to water and releases heat. Heat control methods were adequate. Electrolysis also liberates a lot of energy. The oxyhydrogen output is adjusted to meet the demands of internal combustion engines. The anode received electricity from a 12 V battery, which was then transmitted to the cathode through the electrolyte. The electrolytic glass chamber included everything needed for ingredient delivery and oxyhydrogen generation. When an oxyhydrogen generator was mounted in an engine and no changes were made to the engine assembly, the generator created gas as a by-product. The majority of the gas produced was produced by electrolysis of varied molar concentrations of aqueous catalyst. In this investigation, aqueous sodium hydroxide solutions are used as electrolytes. A semipermeable membrane that is submerged in electrolyte serves to further isolate the anode and cathode electrodes. It is a salt that is made up of the ions sodium and hydroxide, among other components. The use of sodium hydroxide in the production of hydrogen results in increased hydrogen generation rates and lower operating temperatures. The anode received power from a battery, which was then passed on to the cathode through the electrolyte. It was determined that the positively charged anodes were effective in dissolving the water molecules contained in the electrolyte, allowing for the discharge of oxygen and hydrogen gases under the surface of the reactor's upper surface.  Table 2 lists the characteristics of basic fuel gasoline, ethanol, and oxyhydrogen.

## 3. Experimental Details

The nanocoated engine used in the test was constructed in accordance with the parameters that are investigated. It was determined that this study would be conducted using a spark-ignition engine with a compression ratio of 8.5 : 1 and a maximum output of 4.5 kW at 3600 rpm, a single-cylinder four-stroke air-cooled engine. The engine was ready to run after injecting a regulated amount of oxyhydrogen into the air intake manifold and mixing it with fuel and air. Hydrogen's main function is to enrich the reaction, whereas oxygen's primary function is to assist the oxygen enrichment process. This research examined the performance and emission characteristics of ethanol blends and oxyhydrogen utilizing a single-cylinder four-stroke air-cooled SI engine with an incremental load. By mechanical loading, the incremental load was altered.  Figure 1 depicts a schematic representation of an oxyhydrogen and ethanol mix being used in a small gasoline engine.

On the analysis of emission measurement, Crypton 680 series Analyser was used for this research. It is a completely microprocessor-controlled exhaust gas analyser that uses nondispersive infrared (NDIR) techniques. The unit measures CO, CO_2_, and HC. A further channel is provided utilizing an electrochemical measurement of oxygen and chemical sensors used for nitrogen oxides. It has a response time of 10 seconds to 95% of the final reading under operating pressure of 750 to 1000 bar. It operates at a minimum flow rate of 5 litres/min. The technical details of Crypton 680 emission analyser are tabulated in Table 3.

After starting the engine with gasoline, it was subjected to a series of tests until steady-state working conditions were obtained. We examined thermal efficiency, SFC, hydrocarbon, carbon monoxide, and nitrogen oxide emissions. The test runs were conducted using weights proportional to the load's weight. Similarly, when ethanol-blended gasoline with oxyhydrogen enrichment is utilized, similar processes are followed. The ethanol was tested at three different concentrations of 10%, 15%, and 20%, and oxyhydrogen was supplied at a rate of 0.07 g/sec. The air pressure was 1.013 bar at the time of the experiment, and the temperature was about 30°C. To increase precision, each experiment collected all available quantifiable data and computed the mean values. An experimental study was carried out on a gasoline engine with a nanoparticle coating on the piston. 10%, 15%, and 15% ethanol blended with gasoline fuels are used to produce tertiary fuel blends, along with 0.07 g/sec oxyhydrogen injected on trials. On experimental readings, LHRG100 is denoted for the pure gasoline on the LHR gasoline engine. LHRHHOE10 refers to 10% of ethanol and 90% of gasoline blend on volume ratio along with 0.07 g/sec addition of oxyhydrogen on LHR gasoline engine. LHRHHOE15 refers to 15% of ethanol and 85% gasoline blended on a volume basis along with 0.07 g/sec addition of oxyhydrogen on LHR gasoline engine. Similarly, LHRHHOE20 is denoted for 20% of ethanol blended with gasoline along with 0.07 g/sec addition oxyhydrogen.

## 4. Results and Discussion

### 4.1. Effect on Brake Thermal Efficiency

The change in BTE as a function of load is shown in Figure 2, while the combination of oxyhydrogen and ethanol resulted in enhanced combustion, as previously indicated. At full load, the maximum thermal efficiency of oxyhydrogen and ethanol is increased to 19% and 24.8%, respectively, on 15% and 20% blends, showing a substantial performance improvement. Ethanol allows combustion to be completed more quickly. The cycle demonstrates features closer to ideal constant volume combustion and an increase in efficiency [38]. This enhancement occurs as a consequence of higher hydrogen flame velocity and a more diverse spectrum of flames in an oxyhydrogen engine, resulting in a more powerful engine. The combustion rate is decreased when an engine is tested without oxyhydrogen under different load situations. However, oxyhydrogen significantly enhanced the rate of combustion, resulting in an improvement in thermal efficiency.

Additionally, ethanol and gasoline have a lower stoichiometric ratio. It allows the combustion of a larger mass of fuel with the same amount of air. At all loads, oxyhydrogen injection with ethanol mix increased thermal efficiency by 9% to 32% as compared to the LHR gasoline engine. This is caused by stratified charges in the vicinity of the spark plug. The rest of the area is filled by the lean mixture, resulting in a greater combustion rate than when the engine is tested using just gasoline [5]. As a result, oxyhydrogen's properties enable full combustion and excellent thermal efficiency in huge amounts. Due to improved vaporization and air-fuel atomization, the LHR coated engine achieves higher thermal efficiency, maintains maximum in-cylinder temperatures, improves combustion efficiency, and maintains a consistent ignition speed. Additionally, the LHR coating reduces the reject rate of the combustion chamber, increasing the power available to generate with a little quantity of fuel, resulting in increased braking thermal efficiency.

### 4.2. Effect on Brake Specific Fuel Consumption

Figure 3 depicts the effects of injecting oxyhydrogen into ethanol-mixed gasoline, as well as the effects of using just gasoline, on brake specific fuel consumption (BSFC) under four different loads and under a variety of environmental circumstances. The particular fuel consumption was shown to be greater in all blend scenarios, independently of the blend state, although the engine load was originally reduced. One explanation for greater fuel consumption compared to other loads is that the oxyhydrogen generator's partial power absorption is more substantial than that of the other loads, according to hypotheses [39]. Furthermore, since ethanol has a smaller heating valve than gasoline, the temperature fluctuations will be depending on the loads. The engine's specific fuel consumption decreases by 5% to 28.78% when oxygen-hydrogen is introduced into the mixture for all load conditions. The effect of oxygen-hydrogen on specific fuel consumption is magnified when the mixture contains ethanol [40]. According to the testing findings, 20% ethanol resulted in a reduction in fuel consumption ranging between 20% and 28.78% when compared to gasoline usage. Greater flame thrust and calorific values were obtained as a result of the addition of hydrogen and oxygen to gasoline, resulting in chaotic mixing of the air and fuel, which resulted in better combustion than what was accomplished with gasoline alone. Because of the LHR coating's efficient thermal barrier, less heat is needed for cooling and outward dispersion, which results in less heat being transferred to gases in the absence of the coating.

### 4.3. Effect on Carbon Monoxide Emission

CO levels in the air are inadequate and are constrained, and they are mainly utilized to produce low-level ozone. The CO emission rate is shown in Figure 4 as a function of the engine load when supplied with an air/fuel mixture including or not oxyhydrogen. CO emissions are determined by the air-fuel mix and combustion efficiency. CO emissions were reduced by operating the engine at its mid-range speed. Ethanol and oxygen were used to enhance combustion and decrease CO emissions. CO emissions may have been decreased via the use of oxygenated chemicals that enhance CO combustion in the cylinder or during postcombustion operations. However, diluting the gasoline may not be the sole method of reducing CO emissions [6].

Increased combustion and lean engine performance due to the ethanol-oxyhydrogen mix led to CO volume percentage reductions of 2.6% to 9.2% and 7.2% to 20% on 15% and 20% ethanol volumes, respectively. However, the lack of carbon in oxyhydrogen significantly reduced CO production, enabling the engine to run at a low load. In terms of chemical attributes, oxyhydrogen is better, exhibiting a broad range of flammability and a higher flame velocity [41]. A mixture of oxyhydrogen and ethanol-gasoline burns entirely and quickly, totally destroying the pure gasoline. CO emissions are also related to the rate of oxyhydrogen flow, which is especially true at low engine speeds. Additionally, the LHR coating increases cylinder pressure, combustion temperature, and air-fuel mixing, as well as increasing oxygen concentration, which enhances the combustion efficiency of fuel blends [32].

### 4.4. Effect on Hydrocarbon Emission

The findings indicate that the amount of hydrocarbons discharged into the environment is inversely related to the engine speed. Gasoline is incompletely combustible, resulting in the existence of unburned hydrocarbons. In the presence of ethanol and oxyhydrogen, unburned hydrocarbon emissions in the exhaust were decreased by 18% at maximum load and 22% at lowest load, as illustrated in Figure 5. Along with oxyhydrogen, it was discovered that the concentration of HC dropped significantly for all loads. With the addition of oxyhydrogen, a higher degree of full combustion and better engine performance was obtained [42]. As a result, percentage reductions in unburned hydrocarbon volume varied between 3% and 18% when volumetric flow rates of ethanol were used. Hydrogen and the absence of carbon in the reaction mixture accelerate the chain reaction.

This is because the chain reaction happens at a faster rate. Oxyhydrogen injection leads to an increase in crevice area. Hydrogen has a faster quenching time than gasoline, which results in a decrease in hydrocarbon emissions. Due to ethanol's high flammability limitations and the comparatively high in-cylinder pressure and temperature produced by the rapid flame velocity, ethanol blends resulted in a reduction in hydrocarbon emissions [6]. This might be due to greater in-cylinder temperatures caused by increased biodiesel vaporization in the presence of the LHR coating, which enhances soot oxidation and reduces unintended fuel accumulation within the engine cylinder. As a result of the increased oxygen given by ethanol mixture, complete combustion occurs, resulting in lower HC emissions.

### 4.5. Effect on Nitrogen Oxides Emission

The amount of NO_X_ emitted increases significantly, as a result of this method of using oxyhydrogen and ethanol. The presence of oxyhydrogen in the combustion chamber increases both the intensity of combustion and the combustion chamber's temperature. The findings indicated that oxyhydrogen increased NOx emissions, especially when the engine was operated at a low load. Nitrogen oxide emissions in the exhaust were found to be 21.5% more than base gasoline at the lowest load when 20% ethanol and oxyhydrogen were added, as shown in Figure 6. However, with oxyhydrogen injection on the ethanol-gasoline mix, the rate of growth was 20% at the maximum load condition. The main reason for this was a higher concentration of oxyhydrogen in the combustion chamber, which raised the temperature and resulted in the generation of NOx [20].

The temperature of the probe and the excess oxygen concentration in the cylinder have the greatest impact on the generation of NOx emissions. When nitrogen chains are subjected to high temperatures, they break down and disintegrate. Following that, these nitrogen bonds mix with the oxygen molecules stored inside the cylinder to create the monotonic form. The rate at which nitrogen molecules react during combustion is also a factor in the production of NOx emissions when the temperature is increased over a certain point. The Zeldovich mechanism and the availability of oxygen undoubtedly influence the kinetics of O_2_ production. The combustion temperature, which increases NOx generation, is another variable that aids in the interaction between N_2_ and O_2_ molecules [31]. There was an increase in NOx emissions for conventional engines operating at low speeds and for LHR engines operating at full load. This is due to the use of larger cylinders and the melting of a thermal layer coated with YSZ in the combustion chamber [34].

### 4.6. Parametric Optimization of Fuel Consumption and Emission by Full Factorial Design

Experimentation is typically utilized during process development to guarantee that the problem is properly handled. In contrast to the usual approach, this strategy anticipates the understanding and effect of an ongoing complex and the multivariable process by examining individual statistical data from distinct trials. Compared to other sorts of investigation, the design of experiments (DOE) is the most widely applied statistical strategy for optimizing findings. Because operating variables influence engine emissions and performance, itis critical to investigate the impact of many operating parameters on performance of engine and emission responses at the same time [43]. The impacts of optimal engine design parameters on the engine performance and emissions were explored using a multiobjective optimization utilizing a genetic algorithm to discover the optimal values of water injection and different hydrogen energy shares [44]. The effects of hydrogen on a gasoline engine were studied using multiresponse optimization. Torque, hydrocarbon emissions, and engine power were the response factors that were optimized [45]. A full factorial design (FFD) is a basic, rigorous strategy for examining the primary and secondary consequences of research. Although this is a constructive design, the rising relevance of a component or the number of variables demands an increasing number of test points. When the levels and number of variables are decreased, a full factorial design is acceptable. The optimal SFC, CO emissions, and HC emissions were determined using a complete factorial design. As parameters, ethanol additive mixtures, and load fluctuation were selected, as well as their three levels. Minitab 19 was used to accomplish the factorial design and analysis.

In the contour plots provided in Figures 7–9, factorial plots are applied to focus on the important influencing components, such as load and ethanol mixes. This study has revealed that load has a good influence on SFC, with the lowest value attained at full load, which is considered to be related to the engine's increased rate of combustion. Additionally, the fuel consumption rises as the blend ratio increases, diminishing the mix's flammability. Typically, it occurs when ethanol is blended with gasoline at a 20 percent concentration.

CO emissions fall as the load increases, with the lowest emissions occurring at maximum load, as represented by the contour map of carbon monoxide emissions. When a 20% ethanol blend is applied, the emissions levels fall owing to the well-oxygenated mixture, which aids in the thorough burning of the fuel. Because plastic fuel includes a larger number of electrical components than regular diesel, emissions increase as the mix ratio increases. It happens as a consequence of poor fuel mixture composition and sprays formation, leading in incomplete combustion. As per the contour plots, the greatest load applied to the engine and the smallest quantity of ethanol mixture have the most impact on the engine's lowest emissions and fuel consumption.

### 4.7. Response Optimization Results

Optimization is a statistical strategy that is utilized to identify the ideal combination of input variable values for a single answer or a group of replies based on a set of input variables. The response optimizer function in statistical analysis software produces an optimal answer and an optimization graphic for variable input combinations. In some circumstances, an interactive optimization graphic may be appropriate.

The results of response optimization are plotted in Figure 10. The lowest blend ethanol ratio at full load is the most effective strategy to obtain the lowest emissions achievable while keeping the lowest fuel consumption values. Due to the higher combustion rate and oxygenated mixture, this step resulted in complete combustion, which is favourable. According to Table 4, the ideal circumstances for attaining this aim are when the engine is totally loaded. The 75% engine load yields minimum SFC of 0.3358 kg/kWh from a gasoline mix containing 20% ethanol, which is the greatest performance feasible from the ethanol and oxyhydrogen fuel combination. 20% ethanol-gasoline fuel combination yields 2.66 (vol %) of carbon monoxide and 235.41 ppm of hydrocarbon emissions at maximum load condition.

### 4.8. Confirmation Test Results

In order to evaluate the full factorial approach and the response optimization outcomes, a confirmation test is performed, which ensures that the trials' results are consistent with obtained data. The complete factorial design and response optimization approach were used to identify the ideal operating parameters for the crucial variables load and ethanol blend in order to achieve the lowest SFC, lowest CO, and lowest HC. The confirmatory experiment was carried out using the ideal parameters of 75% engine load and 20% of ethanol blend in order to minimize fuel consumption while emitting the least amount of CO and HC emissions as possible. The results of the confirmation test show that the fuel consumption is 0.324 kg/kWh, the CO emission is 2.62% on volume, and the HC emission is 229 ppm. The findings of the confirmation experiments deviate by less than 5% from the optimal values derived from the optimized results.

### 4.9. Environmental Impact of Ethanol and Oxyhydrogen on Gasoline Engine

This research is primarily concerned with minimizing hazardous emissions from a tiny gasoline-powered generator, such as CO and HC. Carbon monoxide is harmful to human health because it impairs the blood's capacity of carrying oxygen to and from tissues. Carbon monoxide quickly enters the bloodstream and converts haemoglobin to carboxyhemoglobin (COHb). When carbon monoxide is detected in the lungs, haemoglobin does not achieve a saturation level of 100% oxygen. According to the American Heart Association, COHb levels of 10% induce headaches, 25% cause nausea and weakness, and 35% cause coma or death in otherwise healthy individuals.

Cognitive impairment, psychological distress, and harm to the respiratory system are all associated with hydrocarbon exposure. Hydrocarbon exposure is also associated with cancer and other general health issues. Additionally, there has been an attempt to quantify toxicity. Benzene is one such substance that causes leukaemia in humans and is found in gasoline and crude oil. Additionally, this hydrocarbon has been shown to reduce white blood cell production, depress the immune system, and increase the vulnerability of white blood cells to infection. There is evidence that many plants are harmed by reactive and hydrophobic aromatic chemicals such as benzenes, naphthalene, styrene, or xylene isomers. Additionally, the phototoxicity of pollutants varies according to the stage of plant development.

Our study established that the addition of oxyhydrogen to an ethanol blend increased fuel economy and efficiency. The smaller engine capacity and combustion conduit enable a wider range of flames and a more rapid rate of combustion. Because hydrogen sharing affected the pace at which the fuel burnt, this study resulted in increased thermal efficiency. Other studies, such as this one, demonstrate significant reductions in pollutant emissions such as unburned hydrocarbons and carbon monoxide. This is because ethanol and hydrogen enrichment accelerates the combustion process and enhances the calorific value of the flame.

## 5. Conclusions

Increased population results in increased energy consumption in the automobile industry. Numerous experts are attempting to develop a replacement for fossil fuel products to satisfy the world's enormous energy demands. The scientists have shifted their focus to alternate energy sources such as ethanol and oxyhydrogen to enhance the engine's performance and decrease hazardous emissions. An experimental study was performed on a small gasoline engine with a nanocoated piston fuelled by an ethanol-gasoline mix with oxyhydrogen as an additive. Three different blends of ethanol used with a constant volume of oxyhydrogen were blended with gasoline. The results show that, along with ethanol and oxyhydrogen, brake thermal efficiency improved by 23% and 32% at 15% and 20% blends, respectively, due to the boost provided by higher flame velocity and a more diverse spectrum of flames when utilizing oxyhydrogen and ethanol. The combustion rate of ethanol-gasoline was substantially increased when a combination of oxyhydrogen was added. Fuel usage was significantly reduced from 5% to 28% on a volume basis under different loading circumstances. Carbon monoxide volume reduced up to 3% to 11% on different blends of ethanol as a result of the increased volume of complete combustion. In the presence of ethanol and oxyhydrogen, the concentration of hydrocarbons dropped by 18% at maximum load and 22% at lowest load, due to the enhanced chain reaction induced by hydrogen. The coating technique has proved for enhanced engine power and reduced fuel consumption due to less heat loss. Also, with better combustion temperature at engine chamber, harmful emissions CO and HC are reduced significantly. Nitrogen oxide emissions were 21% higher than base gasoline at the lowest load, owing to an increase in combustion chamber temperature due to coating. Full factorial design was used to evaluate the influence of engine load and ethanol blends from the experimental results. Response optimization has been utilized for examination to achieve the lowest SFC, CO and HC emissions. The optimization results shows that 75% engine load and with 20% ethanol-gasoline blends results in the lowest fuel consumption and lesser carbon monoxide and hydrocarbon emissions.

Ethanol is a sustainable, domestically generated fuel with a higher octane rating than gasoline, allowing it to perform better than gasoline. Ethanol manufacturing offers jobs in rural communities that are in desperate need of employment possibilities. Ethanol is a bioorganic fuel that may be used to replace fossil fuels in transportation. It has the great potential to contribute to the decarbonisation of transportation and improving the environmental performance. The current research may be extended in the future to high-speed SI engines to improve performance and combustion characteristics by doping nanoparticles with gasoline. The numerical analysis may be performed on a SI engine that is powered by another alternative energy source to improve performance characteristics. Additionally, this study may be improved by including exhaust gas recirculation to help reduce NO_X_ emissions and by modifying it to operate in dual-fuel mode.

## Figures and Tables

**Figure 1:** Schematic arrangement diagram of the gasoline engine experimental setup.

**Figure 2:** Study on brake thermal efficiency on nanocoated ethanol-gasoline engine.

**Figure 3:** Study on fuel consumption on the nanocoated ethanol-gasoline engine.

**Figure 4:** Study on carbon monoxide emission on nanocoated ethanol-gasoline engine.

**Figure 5:** Study on hydrocarbon emission on nanocoated ethanol-gasoline engine.

**Figure 6:** Study on nitrogen oxides emission on nanocoated ethanol-gasoline engine.

**Figure 7:** Contour plot of fuel consumption on load and ethanol blend.

**Figure 8:** Contour plot of carbon monoxide on load and ethanol blend.

**Figure 9:** Contour plot of hydrocarbon on load and ethanol blend.

**Figure 10:** Response optimization plot of SFC, CO, and HC.

**Table 1:** Studies on nanocoating materials and thickness.

Sl. no.	Nanocoating material	Coating thickness (*μ*m)	Researchers
1	Zirconia	300	Sivakumar and Bridjesh [29]
2	Zirconia, zirconia + aluminium oxide (ZrO_2_ + Al_2_O_3_) and fused zirconia (40FZA).	500	Abbas and Elayaperumal [30]
3	Al_2_O_3_/8yttria-stabilized zirconia and CeO_2_/8yttria-stabilized zirconia	300	Gnanamoorthi and Jayaram [31]
4	Titanium dioxide (TiO_2_) and yttria-stabilized zirconia (YSZ)	500	Hafiz Liaqat Ali et al. [32]
6	88% of ZrO_2_, 4% of MgO and 8% of Al_2_O_3_.	400	Aydın and Sayın [33]
7	7YSZ, 2% Gd_2_O_3_+ 5% Y+ 93% ZrO_2_, 5% Gd_2_O_3_+ 2% Y+ 93% ZrO_2_	250	Vidyasagar Reddy et al. [34]

**Table 2:** Properties of gasoline, ethanol, and oxyhydrogen.

Fuel properties	Gasoline	Ethanol	Oxyhydrogen	ASTM testing methods
Chemical formula	C_8_H_18_	C_2_H_5_OH	HHO	—
Density at 20°C (kg/m^3^)	764	787	602	ASTM D4052
Molecular weight (g/mole)	113.89	45.92	16.85	ASTM D2502
Net heating value (kJ/kg)	44000	26812	55000	ASTM D240
Autoignition temperature (°C)	256	361	584	ASTM E659
Stoichiometric air-fuel ratio	14.5	9	34	ASTM D5291
Research octane number (RON)	95	107	130	ASTM D2699
Oxygen content wt.%	0	35	33	ASTM E385

**Table 3:** Details of the emission analyser.

Measurement	Range	Resolution	Accuracy	Instrument
Carbon monoxide	0 to 10%	0.01% vol.	±0.03%	Crypton 680 series analyser NDIR technique
Hydrocarbon	0 to 10000 ppm	1 ppm vol.	±10 ppm	Crypton 680 series analyser NDIR technique
Nitrogen oxide	0 to 5000 ppm	1 ppm	±25 ppm	Crypton 680 series analyser chemical sensor

**Table 4:** Parametric optimized results.

Solution	Load	Ethanol	HC fit	CO fit	SFC fit	Composite desirability
1	75.7576	20	235.416	2.66917	0.335759	0.865620

## Data Availability

The data used to support the findings of this study are included within the article.
